This article has been retracted.

# MiRNA-186-5p Exerts an Anticancer Role in Breast Cancer by Downregulating CXCL13

**DOI:** 10.1155/2022/4891889

**Published:** 2022-02-25

**Authors:** Yulong Wang, Shaojun Hu, Hongbin Zhang, Chenxin Zhang, Qixin Lian, Yu Jiao, Yu Zhou

**Affiliations:** ^1^Tumor Subject, Jiamusi University School of Clinical Medicine, Jiamusi, China; ^2^Department of Oncological Surgery, the Second Affiliated Hospital of Qiqihar Medical University, Qiqihar, China; ^3^Department of Oncological Surgery, the First Affiliated Hospital of Jiamusi University, Jiamusi, China

## Abstract

The aim of this study is to illustrate the biofunctions of miRNA-186-5p level in breast cancer (BCa) and to explore the underlying mechanisms. Levels of miRNA-186-5p in BCa tissues and adjacent normal ones were determined. Association of miRNA-186-5p with pathological parameters and prognosis in BCa patients was analyzed. Luciferase assay was conducted for the prediction of the interaction between miRNA-186-5p and CXCL13. Their mutual interaction in influencing the proliferative potential of BCa was finally explored. Results showed that miRNA-186-5p expression was downregulated in BCa cell lines and tissues. MiRNA-186-5p overexpression could attenuate proliferative ability in BCa cells. A direct and negative correlation was identified between miRNA-186-5p and CXCL13. In addition, their mutual interaction was coresponsible for the malignant development of BCa. In BCa patients, miRNA-186-5p level was remarkably associated with tumor size and tumor staging, rather than other pathological parameters. Low level of miRNA-186-5p predicted a poor prognosis in BCa. Downregulated miRNA-186-5p in BCa is linked to tumor size, tumor staging, and prognosis. miRNA-186-5p downregulates CXCL13 by binding CXCL13 3′UTR in BCa cells. Overexpression of CXCL13 can significantly neutralize the inhibitory effects of miRNA-186-5p on BCa proliferation.

## 1. Introduction

The incidence rate of BCa is relatively high, which ranks first in developed countries. In China, it ranks third among female malignancies [1–3]. Although screening and treatment strategies have been greatly improved, new onset of BCa is growing at a rate of about 2 million each year globally [4]. Surgery is preferred, and it can remarkably enhance the 5-year survival in BCa patients. In particular, the 5-year survival in early stage BCa patients undergoing active treatment can achieve 70–95% [5, 6]. Nevertheless, tumor cell metastasis in advanced stage results in the low survival in BCa patients [7, 8]. Hallmarks of early stage BCa contribute to early diagnosis and treatment in a relatively noninvasive way [9–12].

The newly emerged noncoding RNAs, especially microRNAs (miRNAs), provide a new direction in recognizing molecular events during the development of BCa [13, 14]. From the first discovery of miRNAs in 1993, their biological functions have been gradually revealed. Through targeting mRNA 3′UTR, miRNAs regulate the processes of cell proliferation, differentiation, apoptosis, and other aspects [11, 13, 15, 16]. BCa-associated miRNAs have been identified, which contribute to early diagnosis and comprehensive treatment of BCa [17, 18]. By analyzing the downloaded microarray with BCa profiling, miRNA-186-5p is found to be abnormally expressed in BCa cell lines with a relatively strong proliferative potential [18]. MiRNA-186-5p is differentially expressed in tumor samples [19]. Another previous study showed that miR-186 functions as a tumor suppressor via targeting Twist1 in BCa and might serve as a novel target in BCa diagnosis and therapeutics [20]. The interaction between miRNA-186-5p and CXCL13 is also revealed by online prediction. This study aims to uncover the involvement of miRNA-186-5p and CXCL13 in regulating the proliferative ability in BCa.

## 2. Materials and Methods

### 2.1. BCa Patients and Sample Collection

Tumor tissues and adjacent normal tissues were collected from 48 BCa patients undergoing radical resection. They were newly treated patients and did not have metabolic diseases (e.g., diabetes), cardiovascular diseases, and cerebrovascular diseases. Clinical data and follow-up information were recorded. This study was approved by the Ethics Committee of the First Affiliated Hospital of Jiamusi University and was also conducted after obtaining the informed consent of each subject.

### 2.2. Detection of Cell Viability, Cell Formation, and Cell Proliferation

Breast cancer cell lines (including MCF-7, MDA-MB-231, BT474, ZR-75-30, and SKBR3) and MCF-10A (a kind of normal mammary epithelial cells) were cultured at the concentration of 2 × 10^3^ cells per well. CCK-8 assay (Dojindo, Kumamoto, Japan) was performed daily at different time points. After cell culture for 2 h, the OD value per sample was measured via the microplate reader at 490 nm, and the cell activity curve was plotted. Determination of colony formation was done according to the manufactures' instructions of the colony formation assay kit. Cell proliferation was determined by 5-ethynyl-2′-deoxyuridine (EdU) assay, following the protocols of the EdU assay kit (Sigma-Aldrich, St. Louis, MO, USA).

### 2.3. qRT-PCR TRIzol

qRT-PCR TRIzol was used to extract the total RNA. qRT-PCR was performed according to the previously established instructions. *β*-Actin or U6 served as the internal control. The 2^−ΔΔCt^ method was used for the quantitative analysis. Primer sequences are as follows: miRNA-186-5p: forward: 5′-ACACTCCAGCTGGGCAGCAGCACACT-3′, reverse: 5′-CTCAACTGGTGTCGTGGA-3′; U6 : forward: 5′-CGCAAGGATGACACGCAAATTC-3′, reverse: 5′-TATATCACTCTTGCTTCA-3′; CXCL13 : forward: 5′-GTCCAAGGTGTTCTGGAGGTC-3′, reverse: 5′-CCATTCAGCTTGAGGGTCCA-3′; *β*-actin: forward: 5′-CCTGGCACCCAGCACAAT-3′, reverse: 5′-GCTGATCCACATCTGCTGGAA-3′.

### 2.4. Western Blotting

Total protein extracted from the cells was quantified via the bicinchoninic acid method. Protein samples with the adjusted same concentration were separated and then loaded on polyvinylidene fluoride membranes followed by being blocked with defatted milk (5%) for 2 h and subsequently incubated with primary antibodies at 4°C overnight. Thereafter, secondary antibodies were added for further incubation for 2 h followed by bands being exposed via the ECL kit.

### 2.5. Luciferase Reporting Experiment

MiRNA-186-5p mimics/NC mimics and CXCL13-WT/MMD2-MUT were used to transfect cells in plates (24-well). 48 hours later, cells were lysed for the further measurement of the luciferase activity.

### 2.6. Statistical Analysis

GraphPad Prism and Statistical Product and Service Solutions 18.0 were employed for data analysis. The chi-square test was employed for the relationship analysis between level of miRNA-186-5p and pathological indexes of BCa patients. Statistical significance was set as *P* < 0.05.

## 3. Results

### 3.1. Downregulated miRNA-186-5p in BCa Tissues

A total of 48 matched BCa tissues and adjacent normal ones were collected. Results showed that miRNA-186-5p was lowly expressed in BCa tissues (Figures 1(a) and 1(b)). Additionally, in vitro abundance of miRNA-186-5p was downregulated in BCa cell lines, especially MCF-7 and SKBR3 cells. Furthermore, Kaplan–Meier curves were depicted based on the collected follow-up data. Lowly expressed miRNA-186-5p indicated a poor prognosis in BCa. The enrolled BCa participants were assigned into 2 different groups after calculating the miRNA-186-5p levels in BCa tissues (Figure 1(c)). The association of miRNA-186-5p level with age, tumor size, tumor staging, lymphatic metastasis, and distant metastasis in them was specifically analyzed. Above findings suggested that the miRNA-186-5p level was related to tumor size and also tumor staging in BCa.

### 3.2. MiRNA-186-5p Overexpression Attenuated Proliferation of BCa

MiRNA-186-5p overexpression was constructed via miRNA-186-5p mimic in MCF-7 and SKBR3 cells (Figure 2(a)). Proliferative ability in BCa cells influenced by miRNA-186-5p was tested. miRNA-186-5p overexpression resulted in a significant decrease of BCa cell viability from day 1 to 4 (Figure 2(b)). Furthermore, BCa cells with overexpressed miRNA-186-5p showed fewer visible colonies (Figure 2(c)). Besides, EdU-positive rate decreased by transfection of miRNA-186-5p mimic (Figure 2(d)). It is concluded that overexpression of miRNA-186-5p attenuated proliferative ability in BCa.

### 3.3. CXCL13 Bound to miRNA-186-5p

Through bioinformatics analysis online, three predicted consequential pairings with miRNA-186-5p were found in the 3′UTR of CXCL13. Luciferase assay confirmed that miRNA-186-5p overexpression could attenuate the activity of the luciferase in WT-CXCL13 vector, rather than the mutant-type one (Figure 3(a)). Therefore, we believed that CXCL13 was the downstream target of miRNA-186-5p. CXCL13 was remarkably downregulated in MCF-7 and SKBR3 cells overexpressing miRNA-186-5p at both mRNA and protein levels (Figures 3(b) and 3(c)). Converse to miRNA-186-5p, CXCL13 was upregulated in BCa tissues (Figures 3(d) and 3(e)).

### 3.4. MiRNA-186-5p Regulated Proliferative Ability in BCa by Targeting CXCL13

We next investigated the role of CXCL13 in the development of BCa. It is shown that co-overexpression upregulated CXCL13 than those overexpressing miRNA-186-5p (Figures 4(a) and 4(b)). Interestingly, higher viability and colony number were shown in BCa cells with co-overexpressed miRNA-186-5p and CXCL13 (Figures 4(c) and 4(d)). Taken above, CXCL13 overexpression could abolish the inhibitory effects of miRNA-186-5p in BCa cell proliferation.

## 4. Discussion

In recent years, research studies on the molecular mechanisms of BCa development have made great progress. Nevertheless, surgery and chemotherapy are the conventional therapeutic strategies available for BCa patients [1, 5–7]. Owing to the high metastasis rate in the early phase, it often leads to the fact that BCa patients are already in the advanced stage and lose the surgery opportunity for the first time of diagnosis [6, 7]. Expensive costs and drug resistance remarkably limit the application of newly developed biological therapy and targeted therapy [7, 8]. Therefore, the in-depth study of the malignant biological behaviors and the establishment of infiltration and metastasis blockage are necessary to reduce the mortality of BCa [9–11]. Genetic changes are attributed to the malignant phenotypes of BCa, including expression and functional changes of miRNAs [12, 17, 18].

The current study demonstrated that miRNA-186-5p was lowly expressed in BCa tissues than adjacent normal ones. Moreover, its level markedly correlated to the tumor staging and tumor size of BCa. It is suggested that miRNA-186-5p may have an important anticancer role in BCa. Subsequently, to further explore the effect of miRNA-186-5p on the biological functions of BCa, miRNA-186-5p overexpression was established. CCK-8, colony formation, and EdU assay results altogether uncovered that miRNA-186-5p could inhibit the proliferative ability in BCa cells. However, its specific molecular mechanism was still unclear.

A complicated network involving miRNAs, their targets, and relevant pathways helps us to better clarify the molecular mechanisms of BCa [21, 22]. With the continuous advancement of molecular biology technology, detection of miRNA levels, which is convenient, effective and sensitive, provides a guarantee for early diagnosis of tumors [23, 24]. We verified that CXCL13 was the downstream target binding miRNA-186-5p. CXCL13 was detected to be upregulated in BCa samples and was found to be negatively associated with the miRNA-186-5p level. CXCL13 overexpression abolished the inhibited proliferation in BCa cells overexpressing miRNA-186-5p. To sum up, a negative feedback loop between miRNA-186-5p and CXCL13 exerted an anticancer role in BCa. There are still several limitations in our present study. We only performed the in vitro assays to verify the role of miRNA-186-5p in regulating kinds of BCa phenotypes. Lack of evidence in animal studies made this study deficient. In the future, we plan to complete the validation of the above findings in nude mice, thus to further explore the effects of miRNA-186-5p in tumorogenesis of BCa.

## 5. Conclusions

MiRNA-186-5p is downregulated in BCa samples. The level of miRNA-186-5p is correlated to tumor size, tumor stage, and the prognosis in BCa patients. In general, miRNA-186-5p alleviates the malignant development of BCa via negatively regulating the CXCL13 level.

## Figures and Tables

**Figure 1:** MiRNA-186-5p downregulated in BCa tissues. (a), (b) Levels of miRNA-186-5p in BCa and adjacent normal tissues determined via qRT-PCR. (c) Expressions of miRNA-186-5p in BCa cell lines. ^*∗*^(*P*) < 0.05, ^*∗∗*^(*P*) < 0.01, ^*∗∗∗*^(*P*) < 0.001.

**Figure 2:** Overexpression of miRNA-186-5p attenuated proliferative ability in BCa. (a) qRT-PCR detected the transfection efficacy of miRNA-186-5p mimic in MCF-7 and SKBR3 cells. (b) CCK-8 measured the cell viability of MCF-7 and SKBR3 cells transfected with miRNA-186-5p mimics. (c) Relative colony number in MCF-7 and SKBR3 cells transfected with miRNA-186-5p mimics. (d) EdU assay detected the cell proliferation of MCF-7 and SKBR3 cells transfected with miRNA-186-5p mimics. ^*∗*^(*P*) < 0.05, ^*∗∗*^(*P*) < 0.01.

**Figure 3:** CXCL13 bound to miRNA-186-5p. (a) Luciferase activity in MCF-7 and SKBR3 cells cotransfected with miRNA-186-5p mimics and CXCL13-WT/CXCL13-MUT. (b) Western blotting determined the protein levels of CXCL13 in MCF-7 and SKBR3 cells transfected with miRNA-186-5p mimics. (c) The mRNA level of CXCL13 in MCF-7 and SKBR3 cells transfected with miRNA-186-5p mimics. ((d), (e)) Differential expressions of CXCL13 in BCa and adjacent normal tissues. ^*∗*^(*P*) < 0.05, ^*∗∗∗*^(*P*) < 0.001.

**Figure 4:** MiRNA-186-5p regulated cell proliferation in BCa by targeting CXCL13. MCF-7 and SKBR3 cells were cotransfected with NC mimic + NC, miRNA-186-5p mimic + NC, or miRNA-186-5p mimic + CXCL13. (a) Protein level of CXCL13. (b) The mRNA level of CXCL13. (c) Viability from day 1 to day 4. (d) Relative colony number ^*∗*^(*P*) < 0.05.

## Data Availability

The datasets used and analyzed during the current study are available from the corresponding author upon request.
